The article "Hub Gene Screening and Prognostic Modeling of Lung Cancer: An Integrated Bioinformatics Study" was retracted in 2023. Reasons: suspected computer-generated content; unreliable results or conclusions; lack of ethics approval or compliance; missing or withdrawn patient consent.

# Hub Gene Screening and Prognostic Modeling of Lung Cancer: An Integrated Bioinformatics Study

**DOI:** 10.1155/2022/5110683

**Published:** 2022-07-05

**Authors:** Henan Bai, Xiangdong Huang

**Affiliations:** ^1^Department of Oncology, Chifeng City Hospital, Chifeng, Inner Mongolia, China; ^2^Department of Thoracic Surgery, Chifeng Hospital, Inner Mongolia, China

## Abstract

**Background:**

One of the most frequent malignancies is lung carcinoma which poses heavy burden on the global health. The link among differentially expressed genes (DEGs) and lung cancer patients' clinical outcomes was still missing. In this study, we integrated transcriptome data with clinical data to investigate the relationship between them in lung carcinoma patients.

**Methods:**

To begin, DEGs were identified using the Gene Expression Omnibus (GEO) gene expression pattern (GSE180347). Then, these DEGs are being searched in the TCGA database using the DEGs collected in the preceding phase. The Kaplan-Meier plotter was then used to assess the predictive value of these DEGs in patients with lung cancer.

**Results:**

Our study revealed a total of 45 DEGs, 15 of which were up-regulated and 30 of which were down-regulated. These DEGs were mostly enriched in cytokine receptor binding and cytokine activity, according to GO enrichment analysis. These DEGs were mostly enriched in cytokine-cytokine receptor interaction, according to KEGG enrichment analysis. Based on the PPI network, which comprises of 12 DEGs, a major module was discovered. They are mostly interested in cytotoxicity mediated by natural killer cells. Among all 45 DEGs, the mutations of NCAM1 account for the most cases in TCGA database with a percentage above 15%. Among the 12 DEGs in the significant module, higher expression of FAS, GPR29, HAVCR2, and NCAM1 exhibits longer survival time with hazard ratio and 95% confident interval of 0.79 (0.69-0.89), 0.80 (0.70-0.90), 0.71 (0.60-0.84), and 0.73 (0.62-0.86), respectively. However, higher expression of FCGR3A and IFNG exhibits shorter survival time with hazard ratio and 95% confident interval of 1.50 (1.32-1.71) and 1.15 (1.02-1.31), respectively.

**Conclusion:**

Our results demonstrate significant correlation between some DEGs and the survival outcome in lung adenocarcinomas patients, providing a comprehensive bioinformatics study in anticipation of future molecular mechanisms and biomarker studies.

## 1. Introduction

Lung tumor is a malignancy that starts in the bronchial mucosa or glands of the lungs and is one of the most dangerous cancers for people's health and lives [1]. Lung cancer death rates have increased dramatically in many countries during last 50 years [2]. In males, lung cancer has the highest incidence and mortality rate, whereas in females, tumor has the second highest incidence and mortality rate [3]. Despite the fact that the specific causation of lung cancer is unknown, a large body of research supports a strong relationship between long-term smoking and lung cancer [4]. Long-term cigarette smokers have such a 10- to 20-fold higher risk of lung carcinoma compared to nonsmokers, according to existing studies, and the earlier the age of smoke, the greater the incidence of cancer. Moreover, smoke has a detrimental effect not just on one's own health but also on health of others around them, leading to a rise in the incidence of disease among latent smokers [5, 6].

CD274, also known as PDL1, is a ligand that binds to the T-cell receptor PD1 and inhibits T-cell activation by binding to it. PD1 expression has been seen in melanoma and non-small-cell pulmonary cancer [7]. The interplay of PD1/PDL1 is thought to be a way for tumors to evade the immune system. Several checkpoint blockade drugs targeting the PD1/PDL1 interface have been developed in order to enable T-cells to detect tumor cells without being silenced by the tumor [8, 9]. Infiltration is the basic biological hallmark of malignant tumors, and immunological invasion of tumor cells is metastatic [10]. Malignant tumors have the capacity to penetrate and spread, which would be a biological feature. Since it is an invasive cancer, early detection, diagnosis, and treatment are very important in clinical practice. The characteristics of innate immune infiltration and related lung cancer marker genes may provide novel insights into lung disease immunotherapy [11].

In the present study, the mutations of critical genes play an important impact in the common development mechanism of lung cancer and will affect immunotherapy and chemotherapy, as well as the efficacy of medicine [12]. The relationship between differentially expressed genes and the clinical outcomes of lung cancer patients was still demanded to be explained. The sharing of transcriptome data and the development of new bioinformatics analysis tools have enabled us to integrate transcriptome data with clinical data to investigate the relationship between them in lung cancer development. This can help us understand the development of lung cancer from both perspectives and could offer fresh insights into the disease's prophylaxis and management.

## 2. Material and Methods

### 2.1. Data

The gene expression characteristics (GSE180347) have been retrieved from the Gene Expression Omnibus (GEO) dataset (http://www.ncbi.nlm, http://nih.gov/geo) and used as discovery datasets to recognize differential expression in 34 cases with high total immune cell infiltration (PH) and 7 cases with low total immune cell infiltration (PC) (DEGs).

### 2.2. Identification of DEGs

DEGs were identified using R's LIMMA package [13, 14]. Instead, to avoid the appearance of false-positive results, adjusted *P* values (adj *P* value) were produced. DEGs between PH and PC samples were defined as genes with |log2 fold change (FC)| more than 1 and adj *P* value 0.01. IMMPORT (https://www.immport.org/resources) was used to uncover prospective immunotherapy targets by searching for related immune genes.

### 2.3. GO and KEGG Enrichment Analyses

Using the R packages clusterProfiler and pathview, which are designed to automate biological-term classification and enrichment analysis of gene clusters, the DEGs were analyzed for GO (Gene Ontology) and KEGG (Kyoto Encyclopedia of Genes and Genomes) pathway enrichment.

### 2.4. PPI Network Construction

The DEGs' protein-protein interactions (PPIs) were calculated using the search tool for the retrieval of interacting genes (STRING; https://string.embl.de/), which had a confidence score of 0.9 [15]. The PPI network was then visualized using the Cytoscape program (version 3.5.1). Furthermore, with default settings, the molecular complex detection (MCODE) plug-in in Cytoscape program was used to examine the key modules in the PPI network [16].

### 2.5. Survival Analysis of DEGs

Based on the DEGs obtained from the previous step, these DEGs were searched in The Cancer Genome Atlas (TCGA) database using the combinations of keywords. Based on the recovered cases, the Kaplan-Meier plotter (http://kmplot.com/analysis) might be used to assess the prognostic value of these DEGs in lung adenocarcinoma patients.

### 2.6. Statistical Analysis

Continuous normally distributed data are expressed as means ± SDs. All statistical calculations were carried out using SPSS statistical software. Multiple comparisons were analyzed via analysis of variance (ANOVA). *P* values < 0.05 were considered significant.

## 3. Results

### 3.1. Differentially Expressed Genes (DEGs)

DEGs were identified using gene expression profiles (GSE180347), which consisted of 34 cases with tumors expressing PD-L1 and high total immune cell infiltration (PH) and 7 instances with tumors expressing PD-L1 and low total immune cell infiltration (PC). Our study revealed a total of 45 DEGs, 15 of which were upregulated and 30 of which were downregulated (Figure 1 and Table 1). The 15 upregulating genes were CD55, IFNL1, FCER2, CD34, C6, BLK, TLR5, IL11RA, AMBP, PLA2G1B, NCAM1, CR2, TLR10, CCR6, and CCL14 in descending order of log FC. The 30 downregulating genes were STAT1, PLAU, CDK1, IL1A, ISG15, FPR2, TTK, CD209, SH2D1B, FAS, FCGR3A, CSF2, IFNG, MEFV, HAVCR2, PBK, BIRC5, LILRA5, IL1RN, GNLY, GZMH, SPP1, F12, KLRD1, CD70, CCL13, GZMB, ITGB3, CXCL10, and CLEC5A. Of those 45 DEGs, 25 DEGs were identified as immune-related genes (Table 1). Their functions can be classified as antimicrobials, chemokines, cytokines, chemokine receptors, cytokine receptors, BCR signaling pathway, TCR signaling pathway, and so on.

### 3.2. Functional Enrichment Analysis of DEGs

These DEGs were enriched across several aspects, of which the most significant was cytokine receptor binding, cytokine activity, and virus receptor activity. Besides, exogenous protein binding, receptor ligand activity, signaling receptor activator activity, interleukin-1 receptor binding, immune receptor activity, and signaling receptor activator activity were also differently expressed (Figure 2). These DEGs were shown to be enriched in multiple pathways according to KEGG enrichment analysis (Figure 3). The most important one is cytokine-cytokine receptor interaction, hematopoietic cell lineage, and graft-versus-host disease.

### 3.3. Protein-Protein Interaction Network

The PPI network was built using STRING, and the most important modules in the network were identified using Cytoscape software. The protein-to-protein interaction network of DEGs was complicated in the regulation system, as shown in Figure 4. Genes with high degrees were chosen for further investigation. MCODE discovered a substantial module with 12 nodes and 110 edges (Table 2). The module consists of 12 DEGs, including FAS, STAT1, IFNG, TLR10, CSF2, FCGR3A, HAVCR2, CXCL10, GPR29, GZMB, CD34, and NCAM1. Of the 12 DEGs, FCGR3A is the seeded genes and has the largest degree. TLR10 has the lowest degree. The average degree of the 12 DEGs is 30.5 and the average score is 6.95. They are enriched into several KEGG pathways, including natural killer cell-mediated cytotoxicity, allograft rejection, graft-versus-host disease, type I diabetes mellitus, and so on. The identified 12 DEGs were used for downstream survival analysis.

### 3.4. Survival Analysis of DEGs

The total of 45 DEGs obtained from the previous step was retrieved in the TCGA database. Finally, 248 relevant cases were identified. Among them, there were 102 female cases and 129 male cases. Following the period, 79 cases were dead, while 150 cases are still alive, and 2 cases were not reported. Among the 248 cases, the mutations of NCAM1 account for the most; the following are C6, CR2, and TTK. The GZM8 accounts for the least and then comes the SPP1 (Figure 5). As a result, mutations in the NCAM1 gene were by far the most prevalent. The prognostic of 12 DEGs in the most significant module was explored through the Kaplan-Meier plotter (Figure 6). Higher expression of FAS, GPR29, HAVCR2, and NCAM1 in lung carcinoma patients exhibit longer survival time with hazard ratio and 95% confident interval of 0.79 (0.69-0.89), 0.80 (0.70-0.90), 0.71 (0.60-0.84), and 0.73 (0.62-0.86), respectively. However, higher expression of FCGR3A and IFNG in lung carcinoma patients exhibits shorter survival time with hazard ratio and 95% confident interval of 1.50 (1.32-1.71) and 1.15 (1.02-1.31), respectively. Nonetheless, the expression of the other six DEGs (STAT1, TLR10, CSF2, CXCL10, GZMB, and CD34) did not affect the survival outcome of the lung cancer patients.

## 4. Discussion

The DEGs among high and low total immune cell infiltration in lung carcinoma patients expressing PD-L1 were studied in this research. This study is meaningful since transcriptome data (clinical) were integrated for investigating potential value (prognostic) of DEGs between high and low total immune cell infiltrations in lung carcinoma patients expressing PD-L1. This research can be used to better understand the predictive value of differently altered and to develop clinical diagnoses and treatments.

Our research found 45 DEGs, with 15 upregulated genes and 30 downregulated genes. These DEGs were primarily enriched in cytokine receptor binding and cytokine activity, according to GO enrichment analysis. These DEGs were primarily enriched in cytokine-cytokine receptor interaction, according to KEGG enrichment analysis. By attaching to specific cytokine receptors on the cell surface, cytokines execute biological functions [17]. When a cytokine attaches to its receptor, signal transduction mediated by cytokines begins. Transmembrane proteins contain extracellular, transmembrane, and cytoplasmic domains, which make up the vast majority of cytokine receptors discovered thus far. Cytokines have a broad variety of biological features, including trying to promote target cell proliferation and differentiation, improving anti-infection and cell killing effects, promoting or inhibiting the expression of other cytokines and membrane surface molecules, promoting inflammatory processes, and affecting cell metabolism [18]. A significant module was identified based on the PPI network, which consists of 12 DEGs. Natural killer cell-mediated cytotoxicity is where they are usually found. Among all the 45 DEGs, the mutations of NCAM1 account for the most cases in TCGA database with a percentage above 15%. Importantly, NCAM1 was reported to be a CSC marker and a therapeutic target in solid tumors. NCAM1 was also highly expressed in lung cancer.

Among the 12 DEGs in the significant module, higher expression of FAS, GPR29, HAVCR2, and NCAM1 exhibits longer survival time. However, higher expression of FCGR3A and IFNG exhibits shorter survival time. FAS codes for a member of the TNF-receptor family of proteins [19]. This receptor contains a death domain. It has been discovered to have an important function in the physiologic control of cell death as well as the pathology of a number of immune system malignancies and diseases. FAS-AS1 was significantly downregulated in NSCLC cells. FAS-AS1 could also inhibit cell proliferation, migration, and invasion in NSCLC cells. GPR29 is a beta chemokine receptor with a seven-transmembrane structure that is similar to G protein-coupled receptors [20]. The GPR29 gene is only expressed by immature dendritic cells and memory T-cells. HAVCR2 is a member of the immunoglobulin superfamily as well as the TIM protein family [21]. This Th1-specific cell surface protein modulates macrophage activation, suppresses Th1-mediated auto- and alloimmune responses, and promotes immunological tolerance. NCAM1 is a cell adhesion protein that belongs to the immunoglobulin superfamily [22]. During development and differentiation, the encoded protein is engaged in cell-to-cell as well as cell-matrix interactions. The encoded protein regulates neurogenesis, neurite outgrowth, and cell migration during nervous system development. FCGR3A is a receptor for the Fc component of immunoglobulin G that is involved in the removal of antigen-antibody complexes from circulation as well as other reactions such antibody-dependent cellular mediated cytotoxicity and antibody-dependent intensification of virus infections [23]. The soluble cytokine IFNG belongs to the type II interferon class [24]. The cells from both the innate and adaptive immune systems release the encoded protein. The active protein is a homodimer that binds to the interferon gamma receptor, which initiates a cellular response in response to viral and microbial infections. This gene mutation has been linked to an increased vulnerability to viral, bacterial, and parasite infections, as well as a variety of autoimmune disorders.

The advantage of this study was to identify the related genes that can affect the survival of lung cancer. However, some limitations should be acknowledged. First, only one dataset was added in examination, without considering the effect of population heterogeneity among different countries on the results. Second, the lack of verifiable datasets in this study limits the extrapolation of research results. Third, this study is only for the reanalysis of existing data and lacks the support and verification of experimental data. Finally, our findings give a complete bioinformatics study of high and low total immune cell infiltration in lung cancer patients who express PD-L1, which may aid in the knowledge of lung carcinoma formation, prevention, and treatment.

## Figures and Tables

**Figure 1:** Heatmap plots of DEGs in GSE180347.

**Figure 2:** The enriched GO terms of DEGs in GSE180347.

**Figure 3:** The enriched KEGG pathways of DEGs in GSE180347.

**Figure 4:** Protein-protein interaction network of DEGs in GSE180347.

**Figure 5:** Distribution of most frequently mutated genes in TCGA database.

**Figure 6:** Prognostic of the critical DEGs in lung carcinoma patients.

**Table 1:** Immune-related DEGs in GSE180347.

Gene	Name	Synonyms	Chromosome	Category
BIRC5	Baculoviral IAP repeat containing 5	API4|EPR-1	17	Antimicrobials
CCL13	C-C motif chemokine ligand 13	CKb10|MCP-4|NCC-1|NCC1|SCYA13|SCYL1	17	Antimicrobials, chemokines, and cytokines
CCL14	C-C motif chemokine ligand 14	CC-1|CC-3|CKB1|HCC-1|HCC-1(1-74)|HCC-1/HCC-3|HCC-3|MCIF|NCC-2|NCC2|SCYA14|SCYL2|SY14	17	Antimicrobials, chemokines, and cytokines
CCR6	C-C motif chemokine receptor 6	BN-1|C-C CKR-6|CC-CKR-6|CCR-6|CD196|CKR-L3|CKRL3|CMKBR6|DCR2|DRY6|GPR29|GPRCY4|STRL22	6	Antimicrobials, chemokine_receptors, and cytokine_receptors
CD209	CD209 molecule	CDSIGN|CLEC4L|DC-SIGN|DC-SIGN1	19	Antigen_processing_and_presentation
CD70	CD70 molecule	CD27-L|CD27L|CD27LG|LPFS3|TNFSF7|TNLG8A	19	Cytokines
CR2	Complement C3d receptor 2	C3DR|CD21|CR|CVID7|SLEB9	1	BCR signaling pathway
CSF2	Colony stimulating factor 2	CSF|GMCSF	5	Cytokines, natural killer_cell_cytotoxicity, and TCR signaling pathway
CXCL10	C-X-C motif chemokine ligand 10	C7|IFI10|INP10|IP-10|SCYB10|crg-2|gIP-10|mob-1	4	Antimicrobials, chemokines, and cytokines
FAS	Fas cell surface death receptor	ALPS1A|APO-1|APT1|CD95|FAS1|FASTM|TNFRSF6	10	Natural killer_cell_cytotoxicity
FCGR3A	Fc fragment of IgG receptor IIIa	CD16|CD16A|FCG3|FCGR3|FCGRIII|FCR-10|FCRIII|FCRIIIA|IGFR3|IMD20	1	Natural killer_cell_cytotoxicity
FPR2	Formyl peptide receptor 2	ALXR|FMLP-R-II|FMLPX|FPR2A|FPRH1|FPRH2|FPRL1|HM63|LXA4R	19	Chemokine_receptors and cytokine_receptors
GNLY	Granulysin	D2S69E|LAG-2|LAG2|NKG5|TLA519	2	Antimicrobials
GZMB	Granzyme B	C11|CCPI|CGL-1|CGL1|CSP-B|CSPB|CTLA1|CTSGL1|HLP|SECT	14	Natural killer_cell_cytotoxicity
IFNG	Interferon gamma	IFG|IFI	12	Antigen_processing_and_presentation, antimicrobials, cytokines, interferons, natural killer_cell_cytotoxicity, and TCR signaling pathway
IFNL1	Interferon lambda 1	IL-29|IL29	19	Antimicrobials, cytokines, and interleukins
IL11RA	Interleukin 11 receptor subunit alpha	CRSDA	9	Cytokine_receptors and interleukin_receptor
IL1A	Interleukin 1 alpha	IL-1 alpha|IL-1A|IL1|IL1-ALPHA|IL1F1	2	Antimicrobials, cytokines, and interleukins
IL1RN	Interleukin 1 receptor antagonist	DIRA|ICIL-1RA|IL-1RN|IL-1ra|IL-1ra3|IL1F3|IL1RA|IRAP|MVCD4	2	Cytokines and interleukins
ISG15	ISG15 ubiquitin like modifier	G1P2|IFI15|IMD38|IP17|UCRP|hUCRP	1	Antimicrobials
KLRD1	Killer cell lectin like receptor D1	CD94	12	Antigen_processing_and_presentation and natural killer_cell_cytotoxicity
PLAU	Plasminogen activator: urokinase	ATF|BDPLT5|QPD|UPA|URK|u-PA	10	Antimicrobials, chemokines, and cytokines
SH2D1B	SH2 domain containing 1B	EAT2	1	Natural killer_cell_cytotoxicity
SPP1	Secreted phosphoprotein 1	BNSP|BSPI|ETA-1|OPN	4	Cytokines
STAT1	Signal transducer and activator of transcription 1	CANDF7|IMD31A|IMD31B|IMD31C|ISGF-3|STAT91	2	Antimicrobials

**Table 2:** The most significant module in PPI network.

Gene	Degree	Score	Node status
FAS	24	7.418	Clustered
STAT1	28	6.236	Clustered
IFNG	44	7.418	Clustered
TLR10	14	6.000	Clustered
CSF2	40	7.418	Clustered
FCGR3A	46	7.418	Seed
HAVCR2	20	6.806	Clustered
CXCL10	40	7.418	Clustered
GPR29	22	6.806	Clustered
GZMB	26	7.418	Clustered
CD34	32	6.806	Clustered
NCAM1	30	6.236	Clustered

## Data Availability

The data could be obtained from contacting corresponding author.
